# Big Data-Driven Vocational Undergraduate Talent Training and Social Needs Adaptability Analysis and Collaborative Path Mining

**DOI:** 10.1155/2022/8476412

**Published:** 2022-10-10

**Authors:** Qianqian Lu, Lin Zhang, Chunlei Lin

**Affiliations:** ^1^Administrative Office, Zhejiang Guangsha Vocational and Technical University of Construction, Dongyang 322100, China; ^2^Personnel Department, Zhejiang Guangsha Vocational and Technical University of Construction, Dongyang 322100, China; ^3^Department of Education and Engineering, Zhejiang Guangsha Vocational and Technical University of Construction, Dongyang 322100, China

## Abstract

Aiming at the problem of mismatch between talent cultivation and social demand in the process of undergraduate education, this paper proposes a big data-driven method of adaptability analysis and collaborative path mining between vocational undergraduate talent cultivation and social demand. Starting from the big data-driven vocational undergraduate talent training and social needs, this paper points out the problems existing in the current social needs and puts forward the basic framework of vocational undergraduate talent training mode. Secondly, the clustering model of talent training and social demand is analyzed, and the clustering mining method is proposed. Finally, the big data-driven personnel training and social adaptation mining analysis, in their own ability and social needs adaptability analysis, the basic adaptation accounted for a higher proportion. Professional competence has a higher trust value in cluster analysis. Today's social employment situation is becoming more and more severe, and how to enhance the quality of profession undergraduate students has become one of the theoretical and practical issues worthy of attention in China's colleges at this stage. The talent training model of colleges and universities is closely in route with the demands of society, and the problem of student hire is prominent. Therefore, this paper proposes a student employability training program that combines the elements of student employability through social needs research.

## 1. Introduction

This paper discusses how to cultivate innovative accounting talents in applied undergraduate colleges from four aspects: course content, teaching methods, examination system, and teaching staff, so as to provide an opportunity for the growth of accounting majors in applied undergraduate colleges. Use the industry entry concept to cultivate high-quality and innovative accounting talented people that meet the demands of society. Let the professional construction, teacher training, and education reform of applied colleges jointly promote and innovate [1]. Based on big data, this paper puts forward the merit and defect of the present university teaching methods from the current situation of vocational university reform to the application of modern teaching technology to deepen the “reform of vocational university education which is imperative.” It puts forward modern educational technology countermeasures and deepens the reform of vocational education in colleges and universities. The experiment research results indicate that in the context of the rapid growth of this era of large data, the dissemination and promotion of higher education also require every teacher and student to need innovative ideas, positive thinking, and challenges [2]. The development of economy and informatization has made higher demands for accountants' ideological background, professional theoretical knowledge, business management skills, and comprehensive quality. The traditional way of cultivating accounting talents at the undergraduate level can no longer meet the needs of social development. To this end, application-oriented undergraduate colleges should focus on connecting talents and personnel training goals, serving regional economic development, and innovating the school-enterprise cooperation talent training accounting model [3]. The growth of the times needs the company to have a large number of e-commerce innovation and entrepreneurial talents. The applied education model of innovative and entrepreneurial talented personnel is strongly influenced by the Internet. Reform to suit the growth and needs of today's community. To this end, within the framework of integrating business education, school-enterprise cooperation, and cooperative education, a three-level advanced education model for cross-border e-commerce innovative and entrepreneurial talented person is proposed [4]. The first is to establish a leading mechanism for collaborative innovation of large data analysis and request the talented personnel in colleges and universities; the second is to build a platform for it, and finally, to establish a talent practice base. It aims to cultivate applied talents with large data analysis capability and technological innovation capability to satisfy the remand of economic and social development in the era of big data [5]. Using interview method, questionnaire survey method, statistical method, comparison method, and other research methods, the study reviews the present situation of key teachers and courses of Taekwondo in colleges and universities in Liaoning Province. Through research and analysis of the present circumstances and social needs of talent cultivation, this article aims to provide some preliminary theoretical suggestions and references for the cultivation of Taekwondo undergraduate majors in Liaoning Province [6]. A questionnaire survey was used to compare the social adaptability of professional athletes and students majoring in physical education and to reveal the key factors predicting social adaptability. People with higher education (including athletes and students), male subjects, rural people, or people who have achieved good results in competitions have better social adaptability. Education level can predict different dimensions of social adaptability [7]. The implementation of gifted education in general education is the basic idea of the ““generalist” + “specialist”” education model, which enhances students' social adaptability and professional adaptability. On this basis, a relatively stable standard has been established according to social needs, the needs of discipline development, the school's running direction, school-running conditions, inheritance and training needs, and three professional talent training modes are adopted: basic research, management, and applied technology. Diversified training models focus on cultural characteristics [8]. The short-term forecast analysis of the supply and demand of undergraduate experimental majors in Liaoning Province shows that 105 experimental majors are mainly based on higher vocational education, connected to the secondary industry, and basically compatible with the regional industrial structure. The scope of the 15 experimental professionals in the target year is more or less, and there are relatively few experimental majors related to regional strategic emerging industries. College ought to slightly improve or decrease the enrollment scale, strengthen general education, improve the adaptability of talent training, provide talent support for the growth of pinhead and medium-sized companies, and effectively promote the growth of pinhead and medium-sized companies [9]. Through the introduction of reinforcement cases such as reinforced concrete structures, steel structures, and masonry structures, professional analysis and case analysis are carried out. The research framework of the engineering training platform is built, the teaching content is designed, the textbooks are prepared, and the approaches and strategies for cultivating and improving professional quality and comprehensive quality are provided for the undergraduate engineering level [10]. The structure of social security majors in economic and financial institutions should be combined with the characteristics of financial management colleges. Part of the content clarifies the professional development goals and talent training model, builds a scientific professional talent training platform, establishes a curriculum system that meets the needs of business, management, and social security, and ensures that the professional talent training plan meets the needs of social development [11]. Starting from a clear school-business orientation, that is, the cultivation of applied innovative talents, starting from the “National Standards for Business Teaching Quality” in the “National Standards for the Quality of Undergraduate Education in Colleges and Universities,” to enhance the cultural awareness of innovative talents in the application and analyze the difficulties of corporate talent culture. The majors and typical cases of newly built undergraduate colleges and universities in 8 regions select the talent training path colleges and universities should follow [12]. Through the analysis of the concept of “cooperative education,” the necessity of jointly carrying out “eugenic training” in application-oriented licensing projects is finally proposed, and the idea of “cooperative education” is proposed [13]. Cultivating applied talents is an inevitable requirement for the development and transformation of local colleges and universities. It is necessary to establish a talent training system with skill training as the core and both professional ability and professional quality. Through education reform, school-enterprise cooperation, multiparty participation, and multiparty evaluation, we can realize the integration of gifted education and social needs, achieve the goals of gifted education, and achieve a win-win situation for students and teachers. Schools can achieve, and enterprises can achieve [14]. Combined with the practice of program creation and competition consulting, literature analysis, industry research, educational seminars, and project implementation in the field of large data, it provides overhead quality, hierarchical, and scalable collaborative innovation training models for high-level technical talents. In the large data industry, however, the architecture of large data technologies is changing rapidly. Therefore, the talent training mode, curriculum system, and training plan have formed a recursive process of subjective and objective revision. Finally, it establishes a joint training and innovation practice platform for high-level technical talents in the big data industry. The results of the case study show that the model curriculum system training and practice platform is very effective [15].

## 2. Big Data-Driven Vocational Undergraduate Talent Training and Social Needs

### 2.1. Problems Existing in the Training of Vocational Undergraduate Talents to Meet Social Needs

Practical training is very insufficient. Surveys show that graduates are moving very slowly into management positions. Most graduates need 2–3 years of training and mentoring to be competent for the job, which is also not what employers expect. The main reason for this phenomenon is that the practical training in colleges and universities is very insufficient. Most colleges and universities focus on face-to-face teaching, and students study too much theory and miss practical opportunities. Management is a discipline that closely integrates theory and practice; at the same time, the internal and external environments faced by organizations are constantly changing, and it is almost impossible to do effective management work only by learning from books. The training model lacks innovative consciousness. First of all, the current demand for management talents by employers is no longer traditional professional colleagues but compound talents with management, foreign language, and IT skills. However, many universities are still limited to business studies. The education of some technical knowledge and skills is not comprehensive enough for talents. Second, the quick growth of society has driven the continuous growth of some new fields, such as environmental management and information management. However, many colleges and universities do not offer courses and training in this area, and some colleges and universities only offer courses, which leads to a single form and emerging fields. There is a serious shortage of management talents, and it is hard to satisfy the demand of employers. Third, almost no university dares to provide targeted training, but in a disciplined way, adopts the method of comprehensively promoting leading talents, and leaves specific career guidance to the employer, which also leads to the weak characteristics of leading talents. On the one hand, most colleges and universities only provide career counseling and business information for older students. Many students do not know employers before looking for jobs, and there are no internship opportunities. There is certain blindness in the labor market. On the other hand, many companies are unable to provide colleges and universities with timely information on graduate performance. Colleges and universities do not understand the requirements of enterprises for students' academic qualifications and quality, and it is difficult to find a training model suitable for the work situation of graduates, and it is difficult to make targeted adjustments that will not significantly improve the quality of students. The problems in the vocational undergraduate talent training meeting the social needs are defined as follows:

1. The practical education is seriously insufficient;
2. The training model lacks innovative awareness;
3. The connection between universities and enterprises is not good.

### 2.2. Characteristics of Vocational Undergraduate Talent Training for Social Needs

The difference between applied talents and academic research talents is that applied talents have strong practical ability and can apply the knowledge they have learned in real life. Applied talents emphasize what they have learned and can satisfy the demand of the socially talented person—emphasizing that application in practice refers to the association of theory and exercise and mastering theoretical knowledge more related to practice. For undergraduate applied talents, a theory exists because it has practical value and exists for practice. Prominent application means that the controlled expertise must reach the application level, and everything must be based on the actual situation. Since the improvement of applicability should be gradually realized in the process of solving problems, it is necessary to cultivate talents' ability to find and solve problems through practice. Many problems that arise in practical work are unprecedented, with high levels of difficulty and complexity. It is difficult to find exact answers in textbooks or to answer with knowledge from textbooks. Therefore, teachers should be good at discovering and summarizing laws in practice, using rich experience in argumentation and problem-solving, and reflecting the importance of practitioners' comprehensive practical ability and pioneering and innovative ability. Innovation is not only a matter of time but also the ability and basic quality that applied talents should possess. The application of theoretical knowledge and practical technology by applied talents is not simply inheritance but creative application. That is, they have their own ideas and insights on the original basis and improve their ability by constantly learning and solving new problems. Rigorous, scientific attitude and innovative spirit are the basic conditions for applied talents. The cultivation of applied talents puts forward high requirements for college teachers. The applied talents cultivated by excellent teachers will play different roles in the future and will lead colleges and universities to invest more in the structure of colleges in the process of training applied talents. In addition to their own efforts and practice, students' skills are also inseparable from the teacher's personal development and guidance ability. Sometimes teacher guidance can help students make great progress in some aspects of their research. Therefore, the teachers required to cultivate applied talents are very strict, and there are certain standards for the skills of teachers in all aspects. The cultivation of excellent teachers has also become an important part of the cultivation of applied talents. The vocational undergraduate talents are trained according to their social needs, defined as follows:

1. Application in practice refers to integrating theory with practice and mastering more relevant theoretical knowledge for practice;
2. The teaching staff are good at discovering and summarizing laws in practice, using rich experience to reason and solve problems and improving comprehensive practical ability and pioneering and innovative ability;
3. A rigorous, scientific attitude and innovative spirit are the basic requirements for undergraduate professionals;
4. In the process of cultivating basic professional talents, colleges and universities will be more committed to the construction of their own teaching staff.

### 2.3. The Basic Framework of the Talent Training Model of Vocational Undergraduate Colleges

The mission of vocational undergraduates is to promote employable talents for our country. Although they have some similarities with undergraduate colleges in academic research, they are not the same college, and social and economic development places different requirements on them. Therefore, the gifted education model of research-oriented undergraduate universities cannot be imitated or copied, and the professional training of undergraduate gifted education with its own characteristics should be avoided. Integrated with the research backdrop of this study, this paper analyzes the problems existing in my country's undergraduate vocational education talent training mode and believes that training based on adapting to social needs is the most fundamental direction and choice for forming undergraduate vocational education. Vocational schools in our country: Vocational undergraduates have their own reality, and the talent training models are different, but they are different aspects of talent training, and their components and basic characteristics must be the same. Therefore, this paper focuses on the talent training goals and talent training process: gifted education and teacher level assessment, four elements of the gifted education model, undergraduate professional education, gifted education model framework design, in line with social needs (see Figure 1). The actual situation of colleges and universities' development is oriented by students and social needs, to enhance employment ability-oriented, formulate talent training goals that meet the needs, and guide the talent training process, talent training assessment, and teacher team construction. It should also be implemented on the basis of employability. Just like the development of teachers, it should be applied to undergraduate talents. If corresponding guarantees can be provided in order to achieve the purpose of promoting gifted students, it will also ultimately achieve the purpose of improving students' employability.

### 2.4. Cultivation Strategies for Applied Undergraduate Talents Based on Social Needs

At present, one of the most common drawbacks of talent training in my country's higher education is that it emphasizes the imparting of knowledge while ignoring ability training. They have always followed the traditional ability education model, disregarding social needs, working behind closed doors, and educating teachers with their own ideas. As a result, society does not recruit the talent it needs, and students do not have enough opportunities to find suitable jobs—all in all, a big loss. Different from the promotion of academic research talents who focus on research and experimentation, the main content of applied talents is to cultivate students' application ability. The main goal is to optimize the knowledge structure and quality of basic talent training as a whole, integrate work-related learning programs, and promote the cultivation of applied talents with excellent quality and level. To this end, VET teachers should fully understand the concept of giftedness, emphasize skills and knowledge, and especially focus on improving students' practical ability. Teachers' understanding of the concept of applied talent development will invisibly affect others' understanding, and teachers' behaviors will also promote students' progress. Therefore, it is helpful for teachers to understand the concept of training applied talents. Although practical education plays the main part in the cultivation of applied talented people, because most colleges and universities are still in their infancy in the field of practical teaching, many universities have not perfected the practical education evaluation and supervision system. There is no separate internship system when developing an internship program without regard to internship regulations. Therefore, in teacher training, we should not only notice the transfer of professional knowledge but also notice the evaluation and supervision of practical teaching, create practical learning bases, train practical teachers, and actively carry out practical teaching work. Teachers should not only notice the imparting of knowledge and adhere to a set of teaching methods that go against the grain but also pay attention to evaluating their own teaching methods and monitoring learning effects, discovering the shortcomings of their own education system, improving them, and learning from others. In this way, our continuing education can continue to progress, and the development of applied talents can be smoother. Constructing the education and training of applied talents is not only a good environment for teachers to be assured of training but also the education and training system is very important. The ability to effectively cultivate high-level and applied talents depends not only on a comfortable learning environment but also on a perfect training system. To improve the training system, we should first carry out classification and layered training for teachers to achieve the goal of coordinated development of teachers, and there will be no situation where the level is slightly higher. People with lower ranks cannot compete. Second, we should combine practice and theory, not rely too much on theory, and standardize the practice of teachers. “What you get on paper is superficial, and you must do it without knowing it.” In-depth practice is not only conducive to cultivating applied talents but also conducive to cultivating and improving the level of teachers. The third is the standardization of the training system: no rules can be made without rules, reducing the negative impact of personal factors on trainees and promoting standardized management. The fourth is to regularly hold a training or invite experts to give speeches, improve the skills of each teacher, learn from the excellent experience of others, and better guide students to cultivate applied talents as shown in Figure 2.

## 3. Experimental Models

### 3.1. Overview of Cluster Analysis

The definition of cluster analysis is as follows: given a data set *V*{*v*_*i*_|*i*=1,2, ⋯, *n*}, *v*_*i*_ is a data object, according to the similarity or dissimilarity between the data objects *v*_*i*_, the data set {*v*_*i*_|*i*=1,2, ⋯, *n*} is divided into *k* groups *C*_*j*_(*j*=1,2, ⋯, *k*), and satisfy the following:

(1) $$\begin{array}{c} C_{j}\left|j=\left\{1,2,\cdots ,k\right\}\right.\text{,}\\ C_{j}\subseteq V\text{,}\\ C_{i}\cap C_{j}=\emptyset \text{,}\\ U_{i=1}^{k}C_{i}=V\text{.} \end{array}$$

This process is called cluster analysis, and*C*_*j*_(*j*=1,2, ⋯, *k*) is called a cluster (class).

Given a dataset *V*{*v*_*i*_|*i*=1,2, ⋯, *n*}, *v*_*i*_ is a data object, in the light of the resemblance or dissimilarity between the data objects *v*_*i*_, the dataset {*v*_*i*_|*i*=1,2, ⋯, *n*} is partitioned into *k* organization *C*_*j*_(*j*=1,2, ⋯, *k*), and satisfy *C*_*j*_|*j*={1,2, ⋯, *k*}、*C*_*j*_⊆*V*、*C*_*i*_∩*C*_*j*_=∅、*U*_*i*=1_^*k*^*C*_*i*_=*V*.

### 3.2. Cluster Analysis Algorithm

Assume that the constraint index data of the first level is set as timeliness I, and there are *i* constraints index data at this level, namely *I*_*i*_, and *n* second-level constraint index data are generated from the *i* indicators expressed as follows:

(2) $$\begin{array}{c} I_{i}=\left\{I_{i,1},I_{i,2},\cdots ,I_{i,n}\right\}\text{.} \end{array}$$

The correlation test and analysis of the constrained index data are carried out, and the correlation coefficient between the index data is obtained as follows:

(3) $$\begin{array}{c} r=\frac{cov\left(i,n\right)}{\left|\sqrt{i+n}-1\right|}\text{.} \end{array}$$

In formula (3), cov (*i*, *n*) represents the covariance between the two index data. If *r* is greater than the significance level (*r* > *p*), a partial variance test is performed, and the net correlation between the two data is tested by considering whether there are other interference factors in the index. The coefficient of biased variance is expressed as follows:

(4) $$\begin{array}{c} D_{i,n}=\frac{r_{i}-r_{n}r_{i}}{\sqrt{\left(1-r_{i}^{2}\right)\left(1-r_{n}^{2}\right)}}\text{.} \end{array}$$

The sign of the coefficient can reflect the direction change between the index value and the target value, indicating whether the change trend is consistent. The absoluteness of the correlation coefficient reflects the strength of the correlation. The index data that met the two standardized tests were used in the clustering algorithm for preprocessing.

The sign of the coefficient can reflect the direction change between the index value and the target value, indicating whether the change trend is consistent. The absoluteness of the correlation coefficient indicates the strength of the correlation. The index data that passed the two standardized tests were used to preprocess the clustering algorithm.

In the decision-making process, the cluster analysis algorithm has the advantages of convenient operation, simple and intuitive, and easy to understand. Therefore, according to dynamic cluster analysis, the index data is standardized:

In the decision-making process, the cluster analysis algorithm has the advantages of convenient operation, being simple and intuitive, and easy to understand. Therefore, index data are normalized according to dynamic cluster analysis:

(5) $$\begin{array}{c} u_{i}=K_{i,n}\left(I_{i,n}\right)+c^{2}\text{.} \end{array}$$

In formula (5), *K*_*i*,*n*_ is the number of nuclei of the automatic evaluation index, and *c* is the initial agglomeration point of the automatic evaluation index. According to the group gravity analysis method, the fuzzy dynamic equation is obtained, and the specific expression is as follows:

(6) $$\begin{array}{c} J=\frac{k}{2}\underset{i=1,n=4}{\sum }K_{i,n}\left(I\right)u_{i}^{2}\text{.} \end{array}$$

In formula (6), *k* is the value of the cluster center. Determine the objective function by calculating the distance between the evaluation data and the cluster centers:

(7) $$\begin{array}{c} L=\frac{J}{2}\underset{i=1,n=4}{\sum }K_{i,n}\left(I\right)u_{i}^{2}-\eta \text{.} \end{array}$$

In formula (7), *η* is the automatic fuzzy comprehensive evaluation value. After clustering and integrating the obtained data information, the automatic evaluation data fusion clustering expression is obtained:

(8) $$\begin{array}{c} L=\frac{J}{2}\underset{i=1,n=4}{\sum }K_{i,n}\left(I\right)u_{i}^{2}-\underset{I=1}{\sum }\eta \phi_{i}\text{.} \end{array}$$

In formula (8), *ϕ*_*i*_ is the fuzzy synthesized assess value of the *i*-th optimal scheme. According to the automatic evaluation data fusion method, the output fusion data information is expressed as follows:

(9) $$\begin{array}{c} E=\frac{J}{2}\sum T-\underset{I=1}{\sum }\eta \phi_{i}\text{.} \end{array}$$

On this basis, the construction of the constraint parameter model can be completed, and then the automatic analysis model can be obtained. The estimation formula of automatic evaluation is transformed into the least square solution as in the following formula:

(10) $$\begin{array}{c} R=\sum TE-\underset{i=1}{\sum }\eta \phi_{i}+f\left(t\right)\text{.} \end{array}$$

The time point for evaluating the distribution of big data is represented by *f* (*t*). The synthetic blur magnitude for automated evaluation is calculated using (10):

(11) $$\begin{array}{c} U=\underset{n=1}{\sum }R•w-\underset{i=1}{\sum }\eta \phi_{i}+T\text{.} \end{array}$$

Among them, *w* is the automatic evaluation dynamic blur weight value. The similarity of the evaluation index distribution is solved by using the fuzzy closeness filling method, and the specific expression is as the formula:

(12) $$\begin{array}{c} Y=\underset{n=1}{\sum }R•w+U\sqrt{\lambda }\text{.} \end{array}$$

In formula (9), is the membership degree of each evaluation level. Calculate the factor score coefficients of all subsequences for each sample in the evaluation index data set by the common factor analysis method:

(13) $$\begin{array}{c} x=\underset{i=1}{\sum }UY_{i}^{2}-\frac{T\sqrt{\lambda }}{2}\partial \text{.} \end{array}$$

In (13), is the priori distribution probability of the evaluation. The linear feature fusion way is used to be aware of the fusion of the mean value of the allocation probability of the evaluation index, and the specific expression is obtained as follows:

(14) $$\begin{array}{c} v=\frac{T\sqrt{\lambda }}{2}\partial +\sqrt{m}\sum b_{i}•t+\frac{x_{i}}{Y}\text{.} \end{array}$$

### 3.3. Improved Cluster Analysis Algorithm

First, the sample space is divided into grid cells. The division process is as follows: define the value range of the data space in the *i*-th dimension as (*I*_*j*_, *h*_*j*_), *i* = 1,2, ... , *n*, and use formula (15) to divide it into *p* equal lengths, left closed and right open disjoint interval.

(15) $$\begin{array}{c} \delta_{i}=\frac{\left(h_{i}-I_{i}\right)}{p}\text{.} \end{array}$$

The data space is divided into *p*^*n*^ disjoint grid cells of equal size. The jth array element in the *i*-th dimension is obtained by the following:

(16) $$\begin{array}{c} I_{ij}=\left[I_{i}+\left(j-1\right)\delta_{i},l_{i}+j\delta_{i}\right]\text{.} \end{array}$$

The density and density threshold of each grid cell are then calculated, and high-density grid cells and low-density grid cells are distinguished based on the density threshold. The density threshold is defined as follows:

(17) $$\begin{array}{c} Minpts=\frac{{\left[\sum_{i=1}^{N}Denc{\left(C_{i}\right)}^{2}\right]}^{1/2}}{N}\text{,} \end{array}$$

Denc(*C*_*i*_), *i* = 1, 2,…, *n* is the decreasing order of mesh density, if Denc(*C*_*i*_) and Denc(*C*_*i*_+1) have significant jumps, then *N* = *i*.

This paper adopts the document frequency method based on statistical thinking. Not only the frequency of the word appearing in the text but also the frequency of the word appearing in the text collection, the number of texts in the text collection containing the word, that is, the frequency of the document appearing. The higher the value, the weaker the word's ability to recognize the text, the lower the importance, and the lower the weight should be. Feature location weights are computed using the classic TF-IDF method. The formula for calculating the weight value of feature *T*_*i*_ in text *D*_*j*_ is as follows:

(18) $$\begin{array}{c} TF-IDF\left(T_{i},D_{j}\right)=TF\left(T_{i},D_{j}\right)*\frac{\left|D\right|}{\left|DF\left(T_{i}\right)\right|}\text{.} \end{array}$$

*T*_*i*_ represents a feature, *D*_*j*_ represents the text it is in, *TF*(*T*_*i*_, *D*_*j*_) represents the frequency of feature *T*_*i*_ in text *D*_*j*_, given as word frequency |*D*| represents the total number of texts in the sentence, and |*DF*(*T*_*i*_)| is the feature element. *T*_*i*_ is the number of texts, that is, the frequency of documents. The higher the frequency (word frequency) of the feature element *T*_*i*_ in the text *D*_*j*_, the more representative the content of the text*D*_*j*_, the higher the frequency (document frequency) of the feature element in other texts of *T*_*i*_, the less representative of the content of the text *D*_*j*_.

The greater the frequency (word frequency) of feature item *T*_*i*_ in text *D*_*j*_, the more representative the item is for the content of text *D*_*j*_, and the greater the frequency (document frequency) of feature item *T*_*i*_ in other texts, the more important it is to the content of text *D*_*j*_. Not representative.

## 4. Big Data-Driven Vocational Undergraduate Talent Training and Social Needs Adaptability Analysis and Collaborative Path Mining Analysis

### 4.1. Analysis of the Present Circumstances of Society's Demand for Talents

With the transformation of higher education in China to “popularization,” the total quantity of students in colleges has subjoined from 28.31 million in 2018 to 32.853 million in 2020. The rapid expansion of higher education provides opportunities for millions of students. In recent years, the average annual increase of tens of thousands of graduates from traditional colleges and universities across the country. Measured by the employment rate of advertising graduates, the annual employment rate of college graduates is between 70% and 75%, and the employment rate at the end of the year can generally exceed 90%. In recent years, affected by the epidemic, the employment rate of vocational undergraduate students has shown a downward trend.  Figure 3 shows the trend of talent demand in a province in recent years. From the first season of 2018 to the second season of 2018, the number of talents demanded is on the rise, from 232,932 to 325,263; from the third season of 2018 to the third season of 2020 because of the impact of the popularity in the fourth season, the overall trend of decline was substantial, from 325,263 to 139,487; the growth rate from the first season of 2018 to the third season of 2018 was positive, except the fourth season of 2018 to the fourth season of 2020. Except for the positive growth rate in the second season of 2019, the first season of 2020, and the second season of 2020, all other seasons were negative. Therefore, in recent years, due to the epidemic, the talent market has been hit hard, and the market's demand for talents has dropped significantly.

With the transformation of my state's superior education to “popularization,” the total number of students in colleges and universities has subjoined from 28.31 million in 2018 to 32.853 million in 2020. But, owing to the influences of the murrain last few years, the employment rate has decreased. From the third season of 2018 to the fourth season of 2020, affected by the epidemic, the overall trend showed a sharp decline, from 325,263 to 139,487.

With the growth of the state's income and the country's emphasis on higher education, there are more and more vocational undergraduate talents in our country, so the number of employed people increases accordingly. From the first season of 2018 to the fourth season of 2020, the number of people in the supply increased from 200,027 to 311,354; the growth rate fluctuated, except for the fourth season of 2018, the fourth season of 2019, except for the negative growth rate in the third season of 2020 and the fourth season of 2020, the growth ratio of the rest of the quarters was positive as shown in Figure 4.

In Figure 5, the talent supply and demand ratio increased from the first season of 2018 to the fourth season of 2020, from 0.87 in the first season of 2018 to 2.23 in the fourth season of 2020. From the perspective of stages, from the first season of 2018 to the fourth season of 2018, the talent supply and demand ratio was below 1, indicating that the supply of talents was less than the demand for talents, and the talent market was in a state of shortage; from the first season of 2019 to the fourth season of 2020, the supply-demand ratio is above 1, with a maximum of 2.23. The market is in a situation where supply exceeds demand, and there may be many unemployment problems for talents.

In Figure 5 overall, the talent supply and demand ratio increased from the first season of 2018 to the fourth season of 2020, from 0.87 in the first season of 2018 to 2.23 in the fourth season of 2020, indicating that the market is in a situation where supply exceeds demand and talent. There can be a lot of unemployment status issues.

### 4.2. Analysis of Vocational Undergraduate Talent Training and Adaptability to Social Needs

Adaptability to the social needs of vocational students refers to the tendency of training courses to improve the self-efficacy of vocational students through the training process according to changes in social needs and environmental changes. This research takes the vocational undergraduate student group as the research object, adopts the questionnaire survey method, crosses the two dimensions of autonomy and training mode, and processes and analyzes the results of the questionnaire survey. The adaptability of professional students briefly describes and analyzes the impact and level differences of different characteristics on the adaptability of social needs and provides a reference for subsequent undergraduate talent training strategies. The adaptive analysis results of vocational undergraduate students' own skills and social needs are shown in Figure 6. In terms of professional knowledge, 50.31% of the respondents believe that their professional knowledge can fundamentally meet the changing social needs; however, 36.92% still think that professional knowledge can barely meet the social needs, indicating that most vocational undergraduate students believe that mastering the professional knowledge is a necessary condition to meet social needs; secondly, in terms of practical skills, 51.96% of the respondents believe that their practical skills basically meet social needs, which shows that nearly half of the respondents have a positive attitude towards their practical skills, but there are still 31.11% of people who think that practical skills barely meet the needs of society, indicating that some people think that practical skills need to be improved; in terms of quality development, only 5.79% of people think that their quality requirements do not satisfy the demand of social growth, but most people (62.22%) think that their quality development can basically satisfy the demand of social. From the perspective of three aspects of their own skills, vocational undergraduate students generally have a positive attitude towards their own skills assessment, but there are still a small number of respondents who still need to improve and strengthen their own skills.

The results of “Talent Training and Adaptability Analysis to Social Demands” of vocational undergraduate students are shown in Figure 7. The evaluation is based on four aspects: educational goals, curriculum settings, guidance, and enrollment mechanisms. First, in terms of educational goals, 35.78% of the respondents believed that they were barely able to adapt, and 45.34% believed that they could adapt basically, indicating that there is a certain gap between the goals of higher education and university education and the ability to adapt to social needs; in terms of curriculum settings, only 2.56% of the respondents believe that the course study fully responds to social needs, indicating that there is a certain gap between the curriculum settings of vocational undergraduate students and the adaptation to social needs; with regard to mentor guidance and enrollment mechanisms, vocational undergraduate students are trained to meet social needs (10.95% respectively)., 15.23%), indicating that vocational undergraduate students have certain negative views on teacher orientation and certification, instructing that there is still room for improvement in the direction reform of the teaching staff and the admission process.

### 4.3. Mining and Analysis of the Collaborative Path of Vocational Undergraduate Talent Cultivation and Social Demand

The conformity coefficient assesses the conformity of the measuring content of each project of the questionnaire, and this way is most apposite for reliability analysis of approach and view questionnaires. The reliability coefficients of the four levels of individual control point surveys are as Table 1 shows. It can be plainly found in Figure 8 that the *a*-values of the four levels of different survey contents and overall dimensions are all greater than 0.7, indicating that the overall scale and the subitems of each dimension have good internal consistency reliability.

The four dimensions and eleven components of employability, from the four levels of student recognition, enterprise recognition, student self-assessment results, and enterprise evaluation results, determine the average of the above 11 indicators of employability, then the ten components can be seen from Table 2, and they are best divided into three categories.

According to Table 3 and Figure 9, the first category is the ability to properly cope with stress. It was found to have a high degree of recognition, but a low self-rated score of 3.68 and 2.13 for students and businesses, respectively. The second category of talent training elements has a relatively high degree of recognition. Students basically meet the social needs of this employability, but there is still room for improvement. This is a skill area that colleges and students can be good at. Colleges and universities need to develop these different elements of talent training ability, cultivate students' ability, and enable vocational undergraduate students to adapt to social needs. For the third category of talent training ability elements, most of the scores are around 3, and their recognition is relatively low.

## 5. Conclusion

The development of society and economy requires the education and training of vocational undergraduate students, not only to cultivate academic talents who can engage in professional scientific research but also to cultivate applied and compound talents with research and technology development, management, business, and social service capabilities talent. As a result, purely academic training objectives are no longer sufficient to meet changing social and economic needs. It is necessary to classify the training of vocational undergraduate students accordingly in order to realize the dynamic and developmental changes of training objectives combined with the social needs of employment, emphasizing the diversity of training objectives to satisfy the demand of different types of talented people for the growth of society. Preliminarily set the training goals according to the difference between continuing education and gainful employment, and make reasonable positioning from “simple” to “multiple” to ensure the independence of high-level scientists of scientific research talents from the training goals of high-level talents. At the same time, according to changes in social needs, adjust the training objectives and project parameters in a timely manner, realize the diversification of degree types through the analysis of pros and cons, and learn from the advantages and disadvantages of each person. In line with the development path of disciplines, develop characteristic disciplines and professional research fields. The development of the discipline is closely related to economic development through social and economic needs. Based on the goal of running a school, actively develop characteristic disciplines and focus on the development of characteristic majors. Colleges and universities should dare to innovate and seek breakthroughs within the scope of training disciplines according to the needs of emerging industries and industrial development in society. On the other hand, it provides applied professionals for emerging industries and emerging industries for social needs.

## Figures and Tables

**Figure 1:** The basic framework of the talent training model of vocational undergraduate colleges oriented by social needs.

**Figure 2:** Faculty continuing professional development program.

**Figure 3:** Demand for talents in 2018–2020.

**Figure 4:** 2018–2020 supply talent status.

**Figure 5:** Trend of talent supply and demand ratio.

**Figure 6:** Analysis of self-ability and adaptability to social needs.

**Figure 7:** Analysis of talent training and adaptability to social needs.

**Figure 8:** Reliability analysis.

**Figure 9:** Results of collaborative path analysis.

**Table 1:** Four-level reliability coefficient table.

Test dimension	Test items	Student recognition	Corporate recognition	Student self-assessment	Enterprise evaluation results
Professional ability	Professional knowledge	0.923	0.924	0.876	0.883
	Professional technology				
	Communication skills				
General ability	Collaboration and management skills	0.921	0.918	0.892	0.874
	Innovation and entrepreneurship ability				
	Learning ability				
Personal qualities	Correct coping ability	0.982	0.821	0.794	0.776
	Enterprising				
	Sense of responsibility				
Career planning skills	Career-related competencies	0.775	0.792	0.758	0.736
	Knowledge of career options and development				
Overall scale		0.918	0.933	0.895	0.904

**Table 2:** Cluster analysis results.

Case	4 clusters	3 clusters	2 clusters
Professional knowledge	1	1	1
Professional technology	1	1	1
Communication skills	1	1	1
Collaboration and management skills	1	1	1
Innovation and entrepreneurship ability	2	2	2
Learning ability	3	2	2
Correct coping ability	4	3	2
Enterprising	1	1	1
Sense of responsibility	1	1	1
Career-related competencies	3	2	2
Knowledge of career options and development	2	2	2

**Table 3:** Synergy path analysis table.

Classification	Elements of talent training ability	Student recognition	Corporate recognition	Student self-assessment	Enterprise evaluation results
The first sort	Deal with stress correctly	4.11	4.34	3.68	2.13
The second sort	Professional knowledge	4.56	4.79	4.14	3.56
	Professional technology	4.77	4.94	3.89	2.86
	Communication skills	4.24	4.37	4.65	3.89
	Collaboration and management skills	4.34	4.29	4.34	3.46
	Enterprising	4.37	4.57	4.16	3.59
	Sense of responsibility	4.25	4.78	3.89	3.31
The third sort	Innovation and entrepreneurship ability	3.57	2.89	4.27	3.04
	Learning ability	3.98	3.61	4.24	3.65
	Career-related competencies	3.35	3.14	4.35	3.86
	Knowledge of career options and development	3.62	2.89	3.9	3.31

## Data Availability

The experimental data used to support the findings of this study can be obtained from the corresponding author upon request.
